# The Rehabilitation Training Simulation of High Difficulty Movement and Sports Strain Site Based on Big Data

**DOI:** 10.1155/2021/2911025

**Published:** 2021-09-29

**Authors:** Xiaojie Zhang, Zhengda Ma, Yongming Sun, Yanle Hu

**Affiliations:** ^1^Hebei Sport University, Department of Sports Human Science, Shijiazhuan 050041, China; ^2^Hebei Sport University, Department of Winter Sport, Shijiazhuang 050041, China

## Abstract

We study the rehabilitation training of damaged parts of ice and snow sports clock and ensure the physical safety of athletes. The results show that the RBF neural network updates the center, weight, and width of the radial basis function, and the predicted maximum compliance is 99%, and the minimum compliance is 93%. After many analysis times, the prediction results show that the difference between the predicted degree of conformity and the actual results is less than 8%. The RBF neural network is trained according to the risk database of sports injury, and the RBF neural network will output corresponding values to realize sports injury estimation. The experimental results show that the designed model has high precision and efficiency.

## 1. Introduction

Competitive sports have significant training intensity, and high-frequency competitions are widespread. Many high-level athletes will have various injuries due to different training plans and different priorities of various training stages. With the improved competitive level of ice and snow sports in China, athletes' high-intensity and large exercise training is becoming more and more common. Most ice and snow events are skilled racing events, and in training and competition, athletes often have damage accidents [1]. The high incidence of sports injury affects the training and competition of athletes, causes physical injury, directly affects sports life, and creates excellent results for athletes in snow and ice sports. At present, the injury problem of ice and snow athletes has become a crucial reason affecting sports training and performance. Through the exploration and analysis of the epidemiology and causes of sports injury in ice and ice sports athletes, we can further explore, prevent, treat, and reduce the occurrence of sports injury to minimize the harmful effect of sports injury on athletes and provide a theoretical basis for the sustainable development of snow and ice sports in China.

Sports injury is a common problem in athletes' training. In recent years, with the gradual development of the sports field, the competition among athletes is becoming more and more fierce. The long training time of athletes leads to heavy body load, which makes the incidence of sports injuries higher and higher, seriously affecting the athletes' maintenance and improvement of their achievements, and even causes them to leave the stadium prematurely [2]. Therefore, the treatment and estimation of sports injuries have become a key topic in sports research. Skateboarding which originated in the United States, began to develop in the mid-1960s, and its production is related to surfing, so snowboarding is also called winter surfing. Snowboarding is a sport where athletes fix their feet on a snowboard and slide down a snow slope. Sobko et al. [3] proposed a study method for athlete injury rehabilitation based on extensive data analysis, treating injury from a statistical perspective.

Conducting multilayer linear analysis of rehabilitation factors can obtain the relationship between influencing factors and injury rehabilitation. Describing the occurrence law of sports injury and conducting the principal component analysis of injury rehabilitation factors to obtain the direct influencing factors caused by a sports injury can effectively predict the influencing factors of injury rehabilitation. So, it can complete the injury rehabilitation research of athletes. Reid and Chris proposed a research method for athlete injury rehabilitation based on extensive data analysis. The injury was treated from a statistical perspective. In the 1970s, two important figures appeared in snowboarding. Li and others greatly improved people's control and speed when surfing on snow by improving equipment and snowboarding [4].

Through the improvement of the veneer material and fixer by two people, the veneer gradually evolved from the former semitoy entertainment products to actual sports equipment. They were accepted by more people and eventually developed into a real sport. Wang is also recognized as the founder of modern veneers for his contribution to the veneer movement [5]. In the 1980s, snowboarding became popular in America and soon spread to Europe. With the emergence of the modern veneer, the real veneer competition came into being. As the birthplace of snowboarding in America, the first formal snowboarding competition was held in Colorado in 1981 [6]. As a fantastic individual and new sport symbolizing freedom, snowboarding is becoming more and more popular among young people. The number of snowboarding enthusiasts in the world is increasing day by day. At present, organizing competitions approved by the Federation, formulating and supervising the implementation of competition rules, and handling protests and legal issues related to competitions and rules are all the responsibilities of the International Ski Federation (FIS), which was established in 1924 as the world skiing management organization. Its predecessor was the International Ski Committee, established in 1910. After that, it was reorganized based on the International Ski Committee. The International Snow Federation is an international sports organization recognized by the International Olympic Committee and a member of the International Sports Federation [7–9]. With the success of bidding for the Winter Olympics and enhancing China's economic strength, focusing on the requirements of comprehensively and rapidly developing winter events, the winter project has also received substantial financial support from the China Winter Sports Management Center. Guided by economically developed areas, indoor ski resorts are rapidly built across the country to ensure that athletes have training venues in nonsnow seasons and increase participation in national ice and snow sports. The emergence of numerous ski associations has also accelerated the development and popularization of skiing—a new force to promote skiing in China [10].

Before 2008, there were few related types of research in the field of snowboarding in China. With the continuous improvement of the competitive level of snowboarding in China, the outstanding achievements of athletes in international competitions, and the constant attention of the country, researchers have also generated tremendous research enthusiasm, and the related research studies on snowboarding are gradually increasing. The number of publications has increased significantly since 2008. During this period, Chinese snowboarders gradually achieved excellent results in international competitions, and the popularity of snowboarding events increased [11]. 2015 was the year with the most significant number of publications; from 2003 to this year, a total of 21 academic articles were published throughout the year. The sudden increase in the number of publications was related to the success of China's bid to host the Winter Olympics in 2015, and the winter project became a hot project. Correspondingly, scholars are more involved in snowboarding research [12]. Different authors have different choices of research content. According to numerous literature reports, the development status, technical tactics, equipment, theoretical analysis, and psychological research of snowboarding are the main research directions, most of which are subjective descriptions and analyses by researchers. There are few macrostudies. The Chinese literature on snowboarding lacks articles based on macro research data and with theoretical guidance. However, facing the backward development of snowboarding in China, the lack of such articles harms other aspects of snowboarding research [13]. Although there are studies on the biomechanical analysis of technical movements and sports injuries, the number is tiny. Such research can gain insight into skiers and find and solve problems effectively. Scientific research helps athletes train and recover. Therefore, athletes can improve their competition performance.

Because such a research content is a good guide for snowboarding exercise training, this part of the lack of related research will inevitably affect the comprehensive development of snowboarding sport in our country. To avoid issues related to exposure at a particular stage of development, we should actively carry out relevant research and help us achieve a breakthrough in skiing as soon as possible.

## 2. Research Methods

### 2.1. Multilayer Linear Model of Athletes' Injury Rehabilitation

From the perspective of statistics, the factors affecting athletes' injury rehabilitation were divided into external factors and internal factors of athletes, which were input into a multilevel linear model for analysis. When the multilayer linear model processes the factor data of athletes' injury rehabilitation, the regression equation is first established with external factors' characteristic variable data. Then, the dependent variable is represented by the slope and intercept in the equation. The analysis model is obtained by quadratic regression with the characteristic variable of individual internal factors as the independent variable [14]. Suppose there are *s* independent variables *x*1, *x*2..., and *xs* on the internal factors affecting athletes' injury rehabilitation and *t* independent variables *w*1, *w*2..., and *wt* on the external factors affecting athletes' injury rehabilitation. In this case, two models of athletes' injury rehabilitation levels can be established, as shown in formulas (1)–(3).

Level 1:

(1) $$\begin{array}{c} y_{mn}=\beta_{on}+\beta_{1n}x_{1mn}+\beta_{2n}x_{2mn}+\cdots +\beta_{sn}x_{smn}+e_{mn}. \end{array}$$

Level 2:

(2) $$\begin{array}{c} \beta_{0j}=y_{00}+y_{01}w_{1n}+\cdots +y_{0t}w_{tn}+\mu_{0n},\\ \beta_{tn}=y_{t0}+y_{t1}w_{1n}+\cdots +y_{st}w_{tn}+\mu_{tn}. \end{array}$$

In the formula,

(3) $$\begin{array}{c} COV\left(e_{mn1}\mu_{0n}\right)=\left(e_{mn1}\mu_{1n}\right),\\ COV\left(\mu_{mn1}\mu_{mn2}\right)=0,\;n_{1}\neq n_{2}, \end{array}$$

where *β*_0*n*_ represents the rehabilitation intercept coefficient of the *n*th influencing factor independent variable; *β*_1*n*_... *β*_*sn*_, respectively, represent the slope of the regression of the *n*th influencing factor independent variable to injury rehabilitation. Equation (1) shows that the random errors among individuals are independent within the group. The random error obeys the *P*-dimensional normal distribution, and the error terms of external influencing factors and individual internal factors are independent. Because the individual intrinsic factors of *γ*_*st*_ are not random variations, they are called the fixed parameters of the individual intrinsic factors. *x*_*mn*_ and *w*_*n*_ are, respectively, referred to as the predictors of external influencing factors and individual internal factors. *e*_*mn*_ and *μ*_0*n*_,..., *μ*_*sn*_ are the random effects of external factors and individual internal factors, respectively, indicating that the unit measurement error, *σ*2*e*, and *Σ* are the random effect variance of external factors and individual internal factors, respectively.

### 2.2. Research on Injury Rehabilitation Based on Principal Component Analysis

According to the law of occurrence of sports injuries, the principal component analysis method is used to obtain the corresponding matrix for the internal factors affecting the standardization of individual data, calculate the eigenvalues of the matrix and the eigenvalues of the corresponding eigenvectors, and calculate the variance of the principal components from high to low for each contribution rate. These main parameters influence the injury rehabilitation individual intrinsic factors [15]. By calculating the principal component value of the individual internal factors, the proportion of the influencing factors in the total influencing factors can be analyzed, and the importance of the influencing factors to injury rehabilitation can be predicted. There are five indicators among the individual internal influencing factors, *x*1, *x*2..., *x*5, and *n* athletes' individual internal influencing factors' data matrix can be expressed as shown in the following formula:

(4) $$\begin{array}{c} F_{1}=a_{11}X_{1}+a_{12}X_{2}+\cdots +a_{15}X_{5},\\ F_{2}=a_{21}X_{1}+a_{22}X_{2}+\cdots +a_{25}X_{5},\\ \ldots ,\\ F_{5}=a_{51}X_{1}+a_{52}X_{2}+\cdots +a_{55}X_{5}. \end{array}$$

In the formula, *F*_1_ represents the first principal component; {*a*_*st*_} denotes the second principal component; *T* is for the athlete. The sum of the squares of the coefficients of all principal components is 1 to calculate the coefficient matrix of rehabilitation influencing factors, as shown in the following formula:

(5) $$\begin{array}{c} R=\frac{1}{n-1}X^{*}X^{*T}. \end{array}$$

Making |*λI*-*R*| = 0, five nonnegative eigenvalues are obtained *λs*, and by order of magnitude, i.e., *λ*1 ≥ *λ*2 ≥ ... ≥ *λ*5 ≥ 0. *λ*_*t*_ is defined as the variance contribution of the intrinsic factor *F*_*t*_ of the individual, *λ*_*j*_/∑_*s*=1_^5^×100% is the variance contribution rate of the internal factor *F*_*T*_ of the *t* individual, the sum of variance contribution rates of internal factors of the first *Z* individuals, and ∑_*s*=1_^*z*^*λ*_*s*_/∑_*t*=1_^*m*^*λ*_*s*_ × 100% is the cumulative contribution rate of internal factors of the first *Z* individuals. The number of individual internal factors is *Z*. How much to take depends on the specific situation; usually, the sum of the contribution rate is greater than 85% standard. Principal component values of individual intrinsic factors were calculated. The value of the principal component indicates the degree of influence on injury recovery. After determining the number of principal components of individual internal factors, the principal component values of each in vivo factor can be obtained according to the above formula only by requiring the eigenvectors corresponding to each eigenvalue. The proportion of the influencing factors to the total influencing factors can be analyzed, and the importance of the influencing factors to injury rehabilitation can be predicted.

## 3. Analysis of Research Results

### 3.1. Data Source and Experimental Platform

The objects of the study were snow and ice athletes from all regions of the country, including 63% of the second-level national athletes from the track and field sports students of Liaoning, Henan, Shanxi, Jiangsu, Zhejiang, and Shandong sports vocational and technical colleges. The students were divided into five groups for the test according to their grades and achievements. The total number of people surveyed is 1000, including 500 males and 500 females. The athletes participating in the test are between 16 and 25 years old [16, 17]. The experimental platform is statistical software, and HLM software is used for data processing. The athletes' recovery factors were mainly internal factors and individual characteristics, including the athletes' age, gender, grade, personality, and anxiety. The external factors include the time required for athletes' injury rehabilitation, the amount of athletes' rehabilitation exercise, and the amount of nonrehabilitation exercise. Anxiety is the stress level of the recovery process, which is also indicated on a scale of 0 to 6. The amount of rehabilitation exercise refers to the amount of rehabilitation exercise performed by an athlete to maintain their previous fitness. The amount of nonrehabilitation exercise refers to other activities unrelated to professional sports, which is reflected as an uncertainty in terms of time. Athlete's grade refers to the grade of average performance in ordinary times. Personality is an athlete's level of optimism and pessimism, expressed on a seven-point scale. Anxiety condition refers to the athlete's pressure condition. The sex is 1 for males and 0 for females.

### 3.2. Research Results and Analysis

#### 3.2.1. Analysis of Athletes' Injury Rehabilitation over Time

The athletes' recovery conditions in the questionnaire were statistically analyzed to determine whether there were differences due to time and individual differences of athletes. The analysis results are shown in Table 1. *T*-ratio is the ratio of statistical coefficient and standard error. The result of *P* value can estimate the authenticity of the result (which can represent the whole population), and the reliability of the result of *P* value decreases exponentially, df is the small sample statistic, and *χ*^2^ is the significance test index. The variance of the slope of recovery time and the mean intercept of individual athletes indicate that the slope of each athlete is different, and the recovery time of different athletes is not fixed. The variance of the slope also indicates that the recovery degree of each athlete is not synchronous with time, but there is a rule that the longer the recovery time, the better the recovery degree.

#### 3.2.2. Analysis of the Influence of External Factors on Injury Rehabilitation

The analysis results of rehabilitation and nonrehabilitation activities are shown in Table 2. As can be seen from Table 2, the recovery condition is related to the rehabilitation time and the amount of nonrehabilitation exercise performed by the athletes during the rehabilitation period. The results showed that the relationship between rehabilitation and nonrehabilitation exercise and rehabilitation and exercise varied significantly with individual athletes. It can be seen from the calculation that the variance of the individual internal effect of athletes decreases relative to the variance of the previous experiment. It indicates that the newly added influencing factors strengthen the analysis performance and prove that the influence on injury rehabilitation can be explained by the amount of rehabilitation exercise and the amount of nonrehabilitation exercise. Athletes who performed more nonrehabilitation exercise slowed down the progress of rehabilitation. Athletes perform more rehabilitation exercise activities to speed up the recovery progress.

#### 3.2.3. Influence of Individual Internal Factors on Rehabilitation

The influence of individual internal factors on injury rehabilitation is shown in Table 3. As can be seen from Table 3, age is a significant independent variable of the rehabilitation intercept. Older athletes have a relatively low degree of recovery. In terms of gender, it indicates that male athletes have a lower degree of recovery than female athletes. Male athletes performed more rehabilitation exercises in poor recovery status; for female athletes, the more recovery days they do, the more rehab they do. In terms of age, there was a negative correlation between the amount of nonrehabilitation exercise and the degree of rehabilitation in older athletes. There was a positive correlation between the amount of nonrehabilitation exercise and the degree of rehabilitation in younger athletes. The experimental results show that the older athletes complete more rehabilitation exercises than the younger athletes under a higher degree of rehabilitation, and the more the rehabilitation exercises, the higher the degree of rehabilitation. A dataset matrix was established based on five internal influencing factors of 1000 athletes. Statistical software was used to perform principal component analysis on the questionnaire's dataset matrix of individual intrinsic rehabilitation influencing factors. The cumulative variance contribution rate of individual intrinsic rehabilitation injury influencing factors is shown in Figure 1, with age accounting for 55% and gender for 35%. The cumulative variance contribution rate of their two principal components had reached 90%. Since the cumulative contribution rate is greater than 85%, it can be considered that the first two principal components, age and gender, can represent the main part of the data information of the previous five influencing factors, which are direct influencing factors.

The last ten groups of data in the above analysis of 1000 groups were compared with the actual degree of recovery of athletes to compare and test the degree of conformity of principal component prediction. As shown in Figure 2, the maximum and minimum conformity of the predicted results is 99% and 93%. After many analyses, the prediction results show that, as long as the difference between the conformity degree of the prediction and the real result is less than 8%, it can be considered as an accurate and effective prediction. The main influencing factors predicted by this method are less than 8%, which proves that the predicted results fully meet the requirements.

## 4. Conclusions

The occurrence of sports injuries is complex and changeable. To minimize and avoid the occurrence of sports injuries of athletes in ice and snow sports, a motor injury estimation model is constructed via an RBF neural network. It is suggested that, in the future training and competitions, the athletes of ice and snow sports should try their best to master the correct sports skills and methods of ice and snow sports, make complete preparations and fatigue recovery before and after training, prevent excessive fatigue, control the training rhythm and load, and strengthen the muscle strength training of the vulnerable parts. In the case of physical fatigue or injury, it is necessary to extend the preparation activities appropriately. If necessary, stop exercising and have a good rest. In particular, in serious injuries, it is necessary to wait until the body has fully recovered before resuming training. In addition, athletes should strengthen the study of knowledge of injury and strengthen self-protection and prevention consciousness to maximize and effectively reduce the occurrence of sports injuries. The proposed research method of athletes' injury rehabilitation based on extensive data analysis does not investigate too many external factors due to the limited questions in the questionnaire survey. The principal component analysis is only carried out on the internal influencing factors of individuals, without carrying out the principal component analysis on the external influencing factors. Principal component analysis of other external factors is also carried out to make the influencing factors of injury rehabilitation more precise. A comprehensive and effective prediction is a vital direction of the research on athletes' injury rehabilitation in the future.

## Figures and Tables

**Figure 1:** Principal component analysis diagram of the influence of individual characteristics on rehabilitation.

**Figure 2:** Principal component prediction results.

**Table 1:** The effect of the change of rehabilitation time on injury rehabilitation.

External influence factor	Recovery coefficient	Standard error of *r*	*t*-value	*P* value
Intercept coefficient	1.85675	0.16729	11.46	<0.01
Time slope	0.00155	0.00041	3.78	<0.01
External random effect	Variance	df	*χ* ^2^	*P* value
The average intercept of the individual athlete	2.64576	86	6.754	<0.01
Amount of rehabilitation exercise	0.00372	86	1.016	<0.01

**Table 2:** Analysis results of rehabilitation and nonrehabilitation activities.

External fixation effect	Coefficient	Standard error	*t*-ratio	*P* value
Recovery intercept coefficient	1.90806	0.18221	10.46	<0.01
Slope of recovery time	−0.06436	0.00844	−0.62	<0.01
Slope of rehabilitation exercise time	0.00163	0.00068	2.36	0.018
Nonrehabilitation exercise slope	−0.02152	0.03523	−0.62	0.541
Internal effects of individual athletes	0.94413	—	—	—

**Table 3:** Influence of individual internal factors on injury rehabilitation.

External influence factor	Recovery coefficient	Standard error	*t-*value	*P* value
Intercept coefficient	1.75871	0.29374	6.12	<0.01
Internal factor variable	Coefficient	Standard error	*t*-ratio	*P* value
Age	0.04976	0.01756	2.84	0.004
Gender	0.14392	0.37341	0.39	0.006
Identity	−0.00193	0.01798	−0.12	0.914
Character	−0.04352	0.05098	−0.854	0.393
Anxiety	0.03873	0.02874	1.48	0.214
Individual effect intercept	2.27532	921	2.937	<0.01

## Data Availability

The data used to support the findings of this study are available from the corresponding author upon request.
